The article "Speciation on Oceanic Islands: Rapid Adaptive Divergence vs. Cryptic Speciation in a Guadalupe Island Songbird (Aves: Junco)" was published in 2013. Journal: PLoS One.

# Speciation on Oceanic Islands: Rapid Adaptive Divergence vs. Cryptic Speciation in a Guadalupe Island Songbird (Aves: *Junco*)

**DOI:** 10.1371/journal.pone.0063242

**Published:** 2013-05-10

**Authors:** Pau Aleixandre, Julio Hernández Montoya, Borja Milá

**Affiliations:** 1 National Museum of Natural Sciences, Spanish Research Council (CSIC), Madrid, Spain; 2 Grupo de Ecología y Conservación de Islas (GECI), Ensenada, Baja California Norte, Mexico; 3 Center for Tropical Research, Institute of the Environment and Sustainability, University of California Los Angeles, Los Angeles, California, United States of America; Lund University, Sweden

## Abstract

The evolutionary divergence of island populations, and in particular the tempo and relative importance of neutral and selective factors, is of central interest to the study of speciation. The rate of phenotypic evolution upon island colonization can vary greatly among taxa, and cases of convergent evolution can further confound the inference of correct evolutionary histories. Given the potential lability of phenotypic characters, molecular dating of insular lineages analyzed in a phylogenetic framework provides a critical tool to test hypotheses of phenotypic divergence since colonization. The Guadalupe junco is the only insular form of the polymorphic dark-eyed junco (*Junco hyemalis*), and shares eye and plumage color with continental morphs, yet presents an enlarged bill and reduced body size. Here we use variation in mtDNA sequence, morphological traits and song variables to test whether the Guadalupe junco evolved rapidly following a recent colonization by a mainland form of the dark-eyed junco, or instead represents a well-differentiated “cryptic” lineage adapted to the insular environment through long-term isolation, with plumage coloration a result of evolutionary convergence. We found high mtDNA divergence of the island lineage with respect to both continental *J. hyemalis* and *J. phaeonotus*, representing a history of isolation of about 600,000 years. The island lineage was also significantly differentiated in morphological and male song variables. Moreover, and contrary to predictions regarding diversity loss on small oceanic islands, we document relatively high levels of both haplotypic and song-unit diversity on Guadalupe Island despite long-term isolation in a very small geographic area. In contrast to prevailing taxonomy, the Guadalupe junco is an old, well-differentiated evolutionary lineage, whose similarity to mainland juncos in plumage and eye color is due to evolutionary convergence. Our findings confirm the role of remote islands in driving divergence and speciation, but also their potential role as repositories of ancestral diversity.

## Background

As naturally isolated systems, oceanic islands have long served as unique experimental settings for evolutionary biologists [1]–[5]. Insular radiations such as, *Anolis* lizards in the Antilles, *Drosophila* flies or drepanidid honeycreepers in Hawaii, and Darwin’s finches in the Galapagos Islands, have contributed considerably to our understanding of speciation processes [5]–[8]. However, the rates of evolutionary divergence upon colonization of oceanic islands, as well as the relative roles of drift and selection in driving this divergence are still poorly understood [9], [10]. Natural selection can quickly modify morphological traits following colonization of a new island or isolated habitat type as has been shown in mammals [11] and birds [12], [13], yet the rate and magnitude of change can also be slow and depend strongly on the taxonomic group [14], [15]. In turn, some phenotypic traits can rapidly change in some cases [16], [17], yet can also show limited differentiation over millions of years [6]. Moreover, due to the availability of unoccupied ecological niches in the early stages of island colonization, natural selection can give rise to convergent evolution during diversification, as demonstrated by various dramatic examples in groups as disparate as insects and birds [18], [19]. Due to this variability in patterns and rates of phenotypic divergence, inferring the evolutionary history of insular taxa requires a phylogenetic framework that establishes affinities with mainland relatives and an estimate of time since island colonization, as can be obtained by applying a molecular clock to divergence values from neutral molecular markers [14], [15], [20], [21].

The insular form of the North American dark-eyed junco (*Junco hyemalis*) on Guadalupe Island provides a suitable system in which to investigate the relative roles of isolation and selection in the process of evolutionary divergence. The dark-eyed junco is a common and widespread songbird species in North America, and is composed of several geographically structured color morphs [22], [23] (Fig. 1A). One of these is the island junco *Junco h. insularis,* restricted to the island of Guadalupe (Mexico), 257 km offshore from Baja California (Fig. 1B). This insular population shows a pattern of plumage coloration that is similar to that of the pink-sided junco found in the Rocky Mountains (*J. h. mearnsi*) (Fig. 2), yet it differs from it morphologically, showing a larger bill and smaller body size [22], and a very different song to that of mainland juncos [24].

**Figure 1:** Geographic distributions and sampling localities of the different junco populations. **A.** Distribution map of the genus *Junco* showing schematics of main plumage morphs. Lineage abbreviations, clockwise from south, are the following: VOJU (volcano junco *J. vulcani*), YEJU (yellow-eyed junco *J. phaeonotus*), and the following dark-eyed junco (*J. hyemalis*) morphs: GUJU (Guadalupe junco *J. h. insularis*), GHJU (gray-headed junco *J. h. caniceps*), ORJU (Oregon junco *J. h. oreganus*), SCJU (slate-colored junco *J. h. hyemalis*) and PSJU (pink-sided junco *J. h. mearnsi*). Sampling localities for each morph are marked with colored dots. **B.** Relative position of Guadalupe island with respect to the California shoreline. Juncos on the island are restricted to patches of cypress forest on the northern central plateau (dark green) and the few pine areas along the northern ridge (brown). Main junco distribution ranges are delimited by light green areas.

**Figure 2:** Photographs of individual males of the five junco morphs included in the study. **A.** Oregon junco (*J. h. oreganus*), **B.** gray-headed junco (*J. h. caniceps*), **C.** pink-sided junco (*J. h. mearnsi*) **D.** yellow-eyed junco (*J. phaeonotus*) and **E.** Guadalupe junco (*J. h. insularis*). Note the plumage similarity between C and E.

Continental forms of the dark-eyed junco in the United States and Canada diversified recently as the yellow-eyed junco (*Junco phaeonotus*) of mainland Mexico expanded northward following the last glacial maximum [25]. The Guadalupe junco has a dark iris and plumage coloration similar to some other dark-eyed forms, and thus it is widely thought to be part of this recent radiation [22], [23], [26]. If the Guadalupe junco represents a recent colonization of the island by a continental dark-eyed junco, then morphological changes in bill shape and body size would have taken place in just a few thousand years. The rapid differentiation in morphological traits shown by the recently established dark-eyed junco population in San Diego [27] suggests a capability in the group for rapid adaptation, and an increase in bill size is expected on island populations as it increases potential access to a broader range of food resources [28].

Here we use divergence time estimates obtained from mitochondrial DNA (mtDNA) sequence variation to test whether the Guadalupe junco evolved recently following a colonization by mainland dark-eyed juncos (as iris and plumage color suggests), or instead represents a “cryptic”, well-differentiated lineage adapted to the insular environment through long-term isolation, with plumage coloration being a result of evolutionary convergence. To do so, we use mtDNA sequence, morphological measurements and song variables to compare the Guadalupe population (*insularis*) to several continental populations of the dark-eyed junco (including the Oregon junco *J. h. oreganus*, pink-sided junco *J. h. mearnsi* and gray-headed junco *J. h. caniceps*), as well as the yellow-eyed junco (*Junco phaeonotus*) from mainland Mexico (Fig. 2).

## Results

### Genetic Divergence and Diversity

Sequencing of two mtDNA markers in 87 individuals (Table 1) produced 9 haplotypes for the control region (CR), and 7 haplotypes for the cytochrome *c* oxidase *I* (COI) gene, resulting in 14 haplotypes for the concatenated sequence (989 bp). Phylogenetic analysis of the concatenated mtDNA haplotypes revealed the presence of two highly divergent genetic lineages: one corresponding to *insularis* individuals from Guadalupe Island, and one that included all continental dark-eyed and yellow-eyed juncos (Fig. 3A). One individual from Guadalupe Island (showing a typical Guadalupe phenotype) was found to carry mainland COI haplotype “A” (Fig. 3B), suggesting it descends from a female that reached the island relatively recently, yet long enough ago to show some mtDNA divergence, as its control region haplotype (“U”, Fig. 3C) does cluster with the remaining Guadalupe CR haplotypes. The mainland lineage showed a “star-like” pattern consisting of a high-frequency haplotype (“AA”) surrounded by various lower frequency haplotypes, a pattern characteristic of a recently expanded population as previously reported for these populations [25], and one that is not apparent in Guadalupe Island.

**Figure 3:** Mitochondrial DNA haplotype networks of Guadalupe, continental North America and volcano juncos (VOJU). Shown are median-joining networks for the concatenated CR and COI sequences (**A**), COI (**B**) and CR (**C**). Haplotypes are represented by circles, their size proportional to their frequency in the population. Color patterns are as follows: orange – *Junco phaeonotus,* blue tones – continental *Junco hyemalis* (dark: ORJU, light: PSJU, purple: GHJU), green – *Junco h. insularis*. Each branch represents a single nucleotide change, with additional mutations indicated by bars along branches. Numbers in squares indicate nucleotide changes separating the volcano junco.

**Table 1:** Mitochondrial DNA haplotype frequencies in junco populations.

Lineage	N	COI	CR	CR+COI
**ORJU**	22	A (21), U (1)	A (20), M (2)	AA (19), AU (1), MA (2)
**PSJU**	4	A (4)	A (3), M (1)	AA (3), MA (1)
**GHJU**	5	A (5)	A (3), I (2)	AA (3), IA (2)
**YEJU**	24	A (23), O (1)	A (14), E (10)	AA (13), AO (1), EA (10)
**GUJU**	32	A (1), J (6), K (10), L (13), M (2)	T (22), U (1), V (5), W (4), X (1)	TJ (6), TK (9), TL (4), TM (2), UA (1), VL (5), WL (4), XK (1)

Haplotypes for cytochrome *c* oxidase gene (COI), control region (CR) and the concatenated dataset (CR+COI) are denoted by letters, with the frequency of each indicated in parentheses. Lineage codes correspond to continental dark-eyed forms *J. h. oreganus* (ORJU), *J. h. mearnsi* (PSJU) and *J. h. caniceps* (GHJU), yellow-eyed junco *J. phaeonotus* (YEJU) and Guadalupe junco *J. h. insularis* (GUJU).

Genetic divergence based on the concatenated dataset was greater between *insularis* and either continental lineage (1.20% between *insularis* and continental *hyemalis*, and 1.22% between *insularis* and *phaeonotus*) than between both continental lineages (0.07%) (Table 2).

**Table 2:** Genetic distances between the three junco lineages.

CR\COI	DEJU	YEJU	GUJU
**DEJU**	0.31\0.06	0.07	7.72'
**YEJU**	0.58'	0.51\0.08	7.73'
**GUJU**	4.10'	4.35'	0.67\1.34'

Mean number of substitutions for CR (349 bp) are shown below the diagonal and for COI (640 bp) above the diagonal. Lineage abbreviations are as follows: continental dark-eyed junco (DEJU), yellow-eyed junco (YEJU) and Guadalupe junco (GUJU).The marked differentiation of *insularis* with respect to continental lineages is visible in both mtDNA markers. However, the number of nucleotide changes in the CR sequences is lower compared to those in COI, reflecting a lower mutation rate or, more likely, high rates of homoplasy in the control region, as documented in previous studies [29], [30].

Applying a standard clock calibration of 2.1% divergence per million years (Ma) for coding mtDNA genes in passerines [31] to our COI sequences, we estimated the time to the last common ancestor between *insularis* and the continental *hyemalis* forms at 0.58 Ma ago, within the middle Pleistocene. Rate correction using the curve for avian mitochondrial protein coding genes in Ho *et al.* [32] places the divergence time around 0.43 Ma. Isolation-with-migration results from the MCMC runs on IMa2, with a 0.01 mutation rate per site per lineage per Ma for COI sequence data, estimated a divergence time between the continental and island lineages of 0.60 Ma, and considered a migration rate (m) from the continent to the island of 1.6×10^−6^ individuals per year, with no gene flow detected from the island to the continent. Analysis with BEAST 1.7.2 revealed homogeneous substitution rates across branches, and clock rate estimation with a fixed clock model set the clock rate to a mean of 0.023 divergence per site per Ma (SE = 0.0014). Since the distribution of the parameter was not normal, a better estimator of divergence time for the most recent common ancestor between Guadalupe and continental haplotypes is the median time, which was 0.57 Ma (with a mean time of 0.77 Ma, SE = 0.0072).

Genetic diversity was higher in Guadalupe Island than in the mainland populations, even when the recent immigrant to the island was excluded from analysis (Table 3). Nucleotide diversity and haplotype diversity indices on the island were an order of magnitude larger than in the continental populations for the COI sequences (Table 3). The values for the control region show less contrast between island and continent, partly because of the high frequency of control region haplotype T on the island, likely due to homoplasy as higher mutation rates in this region are likely to give rise to the same changes independently in different lineages. F_s_ values are negative and significant for continental dark-eyed juncos for the COI region, consistent with a population expansion as previously reported by Milá *et al.* [25]. The *insularis* lineage, however, does not show a significant pattern of population growth, and F_s_ values are consistent with long-term demographic stability.

**Table 3:** Genetic diversity and demographic history indices of junco lineages.

		COI				CR			
Lineage	N	N Hap.	*h*	*π*	F_s_	N Hap.	*h*	*π*	F_s_
**DEJU**	31	2	0.07±0.06	0.0001±0.0002	−1.24*	3	0.29±0.10	0.0009±0.0010	−0.85
**YEJU**	24	2	0.08±0.07	0.0001±0.0002	−1.03	2	0.51±0.04	0.0015±0.0014	1.53'
**GUJU**	32	5	0.72±0.04	0.0021±0.0015	0.22	5	0.54±0.09	0.0019±0.0016	−1.64
**GUJU (excluding** **immigrant)**	31	4	0.70±0.04	0.0014±0.0011	0.17	4	0.51±0.09	0.0017±0.0015	−0.86

Haplotype diversity (*h*), nucleotide diversity (*π*) and Fs values for the three junco groups (pooling populations): Continental dark-eyed juncos (DEJU), yellow-eyed juncos (YEJU) and Guadalupe juncos (GUJU). The bottom row shows values obtained when excluding an individual that is likely a recent immigrant to the island (see text). *P<0.05.

### Morphological Divergence

The discriminant function analysis of morphological traits shows a clear separation between all three forms (*insularis, hyemalis* and *phaeonotus*), and reflects the overall small size and large bill of *insularis* (Fig. 4). The first discriminant function represents overall larger birds with smaller bills, and the second function corresponds to larger birds with smaller wings (Table 4).

**Figure 4:** Discriminant function analysis of morphological variables from the different junco lineages. *J. h. insularis* (green squares), *J. h. oreganus* (blue squares), *J. h. mearnsi* (blue circles), *J. h. caniceps* (purple triangles) and *J. phaeonotus* (yellow circles). Empty circles represent group centroids. Correlation values between discriminant functions and transformed morphological variables are shown in table 4.

**Table 4:** Standardized coefficients for the first two canonical discriminant functions from morphological measurements.

Variable	DF1	DF2
**LnWing**	−0.218'	0.891'
**LnTail**	−0.418'	−0.240'
**LnCulmen**	0.557'	1.039'
**LnExp.Culmen**	0.123'	−0.957'
**LnDepth**	0.480'	0.067'
**LnWidth**	0.074'	0.070'
**LnTarsus**	0.076'	−0.466'
**(Weight)^⅓^**	−0.631'	−0.237'

Discriminant functions DF1 and DF2 account for 65.7% and 32.0% of the total variance, respectively.

Morphological analysis showed marked divergence in trait mean values between *insularis* and continental forms (Fig. 5). *Insularis* individuals showed significantly smaller mean values for weight, wing length and tail length (weight: *F*_2,104_ = 85.3, *P*<0.001; wing: *F*_2,106_ = 242.7, *P*<0.001; tail: *F*_2,102_ = 155.3, *P*<0.001), yet had larger bills than both mainland forms (bill culmen: *F*_2,108_ = 146.6, *P*<0.001; exposed bill culmen: *F*_2,108_ = 82.5, *P*<0.001; bill width: *F*_2,108_ = 18.0, *P*<0.001 and bill depth *F*_2,108_ = 56.9, *P*<0.001), and an intermediate tarsus length (*F*_1,74_ = 16.9, *P*<0.001 *insularis* vs. continental *hyemalis*). Members of the *phaeonotus* lineage also tend to be larger and heavier than their northern relatives.

**Figure 5:** Differences in morphological trait means among junco lineages. Bars correspond to 95% confidence intervals. Abbreviations correspond to Guadalupe junco (GUJU), continental dark-eyed juncos (DEJU) and yellow-eyed junco (YEJU). Units of measurement for weight are grams, and wing, tail, tarsus and bill variables are in mm.

### Song Divergence

Differences in song structure and note diversity are apparent between the three lineages, with the song of continental *hyemalis* (represented here by the Oregon junco *J. h. oreganus*) consisting of a simple trill, whereas the songs of *phaeonotus* and *insularis* contain a greater diversity of syllables (Fig. 6). A discriminant function analysis of song variables clearly separates the three lineages along the axis of the first discriminant function (Fig. 7), which correlates with increasing frequency range and number of different syllables per song (Table 5). Diversity in *phaeonotus* songs is intermediate between *insularis* and *oreganus* song types, showing less variability and more repetition of syllables than the *insularis* song (Fig. 6). There are significant differences between *insularis* and mainland forms (*hyemalis*+*phaeonotus*) in number of different syllables (*F*_2,29_ = 130.5, *P*<0.001), maximum frequency (*F*_2,29_ = 16.3, *P*<0.001), minimum frequency (*F*_2,29_ = 32.4, *P*<0.001) and number of repeated elements (*F*_2,29_ = 25.7, *P*<0.001).

**Figure 6:** Song spectrograms for representative song types from the three junco lineages. **A.** *J. h. oreganus*, **B.** *J. phaeonotus* and **C.** *J. h. insularis*. Amplitude (y-axis) is given in KHz, and time (x-axis) is in seconds.

**Figure 7:** Discriminant function analysis of song variables for the three junco lineages. *J. h. insularis* (green squares), *J. h. oreganus* (blue triangles) and *J. phaeonotus* (orange circles). Empty circles represent group centroids. See Table 5 for correlation values between discriminant functions and song variables

**Table 5:** Standardized coefficients for the canonical discriminant functions from song variables.

Variable	DF1	DF2
**Number of different syllables**	0.895'	0.074'
**Minimum freq.**	−0.204'	−0.525'
**Maximum freq.**	0.494'	0.379'
**Syllable repetitions**	−0.060'	1.215'
**Song duration**	−0.428'	−0.408'
**Peak freq.**	0.305'	−0.351'

Discriminant functions DF1 and DF2 account for 96.3% and 3.7% of the total variance, respectively.

## Discussion

### Genetic Divergence and Phenotypic Convergence on Oceanic Islands

Our results reveal marked mtDNA divergence between *insularis* and continental junco lineages, supporting the hypothesis of a long history of isolation for the Guadalupe junco. Despite plumage and eye color similarities with mainland dark-eyed juncos, Guadalupe juncos represent a well-differentiated lineage that split from continental forms about 0.5 million years ago, well before the start of the postglacial expansion and radiation that gave rise to the continental dark-eyed juncos in the Holocene [25]. Thus the prevailing hypothesis postulating that the Guadalupe junco represents a recent colonization of a continental hyemalis dark-eyed form [22], [23] can be rejected, in favor of the alternative hypothesis for a case of convergence in plumage color.

The study of insular organisms with molecular tools has revealed numerous cases of evolutionary convergence in many different taxonomic groups, from insects [18] to birds [19], and not just in oceanic islands but also in similarly isolated continental environments organisms, such as cichlid fishes in isolated freshwater African lakes [33]. Convergence often reveals the action of similar selective factors acting in a similar way to modify phenotypic traits in unrelated lineages, providing insight into the specific factors that are important in the early stages of divergence in insular organisms. The convergent plumage color found in the Guadalupe junco and the continental pink-sided junco, consisting of similarly patterned patches of gray, brown and rufous areas, is unlikely to be the result of environment-driven natural selection, given for instance the marked differences in the habitats where each taxon lives (arid cypress forest and scrub in Guadalupe vs. high-elevation conifer forest and alpine meadows in the Rocky Mountains, respectively). However, it could be due to sexual selection acting on plumage color traits through female choice. Plumage pattern may have appeared in the population from standing variation or by a stochastic mutation-order process [34] in which a de-novo mutation could give rise to a similar plumage by chance, and be subsequently driven to fixation through sexual selection. Analysis of plumage patterns across all Junco taxa in a phylogenetic context will be necessary to better understand plumage evolution in the group.

### Genetic Diversity on Guadalupe Island

The relatively high amount of haplotypic and nucleotide diversity within the *insularis* lineage, together with the non-significant F_s_ values, reveal a surprising absence of population bottlenecks in the history of the lineage, despite the necessarily low population sizes juncos there must have experienced. At least during the last 200 years, a feral goat infestation severely reduced the area of suitable junco habitat from at least 780 ha [35] to currently less than 210 ha. Although this anthropogenic reduction in population size could be too recent for diversity to have been lost by drift, our result is inconsistent with the expected diversity loss often detected in small oceanic islands [20], [36]–[42], and indicates that historical effective population sizes (N_e_) have been sufficiently large to maintain variability, at least until recently. Other studies reporting relatively high genetic diversity in insular bird populations correspond to natural colonizations by large flocks or management-driven reintroductions in historical times [43], [44].

Islands can represent refugia for a species’ genetic diversity in cases where habitat destruction or genetic introgression by invasive competitors has affected original diversity in mainland parts of its range [45], [46]. In the case of the Guadalupe junco, this insular population constitutes a repository of ancestral genetic diversity in a species complex that has suffered a widespread loss of genetic diversity across the continent, not because of recent anthropogenic factors, but due to the impact of natural glacial cycles on the historical demography of continental populations [25].

The presence of haplotype “UA” in the *insularis* lineage indicates an event of secondary colonization by at least one mainland female, as supported by the migration rates towards the island population in the coalescence simulations. The phenotype of the individual in question is however indistinguishable from other Guadalupe juncos, suggesting that the nuclear genome has become homogenized through recombination since colonization. Arrival of migratory continental *hyemalis* individuals to the island is probably not uncommon, which combined with the low level of introgression detected here, suggests that premating reproductive isolating barriers might have evolved, as suggested by an interesting sighting by Bryant [47] in the late nineteen-hundreds, who witnessed an Oregon junco (*J. h. oreganus*) being attacked by Guadalupe juncos during a windy day in the pine forest on the northern tip of the island.

### Phenotypic Divergence of the *insularis* Lineage

Our morphological analysis confirmed that *insularis* birds are smaller than mainland individuals, yet have significantly larger beaks. Increased beak size has been previously observed in insular passerines, and is commonly associated with a wider range of food resources resulting in part from a lesser number of competing species [20]. In the case of Guadalupe Island, a potential additional factor driving changes in bill size and shape could be related to feeding on the large seeds within the hard cones of the endemic cypress *Cupressus guadalupensis*. Juncos could have relied heavily on these seeds over at least the last 200 years, a period during which the feral goat infestation severely restricted the juncos’ diet, until the extirpation of the goats just five years ago [48]. Experimental approaches will be necessary to properly test the role of cypress seeds in driving adaptive morphological divergence in Guadalupe juncos.

The song of *insularis* males is also markedly different from that of mainland males. Although divergence from continental song was expected due to the population's long-term isolation, complexity of the long-range song performed by *insularis* males goes against the expected loss of diversity in small islands [49]–[51]. Similarly high levels of song diversity and complexity have been recently reported by Pieplow and Francis [52], for Baird's junco (*Junco phaeonotus bairdi*) in the Sierra de la Laguna Mountains at the southern end of the Baja California peninsula (Mexico), a small “sky island” located more than 300 km away from the nearest yellow-eyed junco population. It remains to be tested whether song types in these isolated lineages represent ancestral levels of diversity since lost in mainland populations, or alternatively, whether diversity could be the product of increased competition for resources and thus increased sexual selection in small areas with restricted resources.

In contrast to the observed divergence in morphology and song, iris and plumage color in the Guadalupe junco are very similar to that of some continental populations, which led most previous experts to consider the insular form as one of the “dark-eyed juncos” [23]. Our genetic results reveal that plumage color in Guadalupe juncos represents a case of evolutionary convergence and that dark eye color seems to have evolved more than once in the complex. Thanks to molecular dating, the lability and often fast evolution of plumage color has been documented in several groups, including orioles [53], wagtails [54], parakeets [55] and warblers [56]. Within the latter group, a recent study of insular forms of the yellow warbler (*Setophaga petechia*) revealed that the color pattern found on the Galapagos Archipelago has evolved at least once more independently on the mainland, rendering plumage color uninformative for reconstructing the evolutionary history of the group [57].

Overall, both drift and selection appear to have played a role in driving the divergence of *insularis*. Divergence in neutral genetic loci suggests the role of drift, yet marked divergence in morphological structures related to feeding (bill shape) and locomotion (wing and tarsi), as well as male song characteristics, strongly suggest the role of natural and sexual selection in driving divergence, as has been demonstrated in other better studied natural systems [58]–[61]. Further research on the adaptive value of these phenotypic traits and their effect on the fitness of individuals will be necessary to fully understand divergence mechanisms in this island system.

### Taxonomic and Conservation Implications

*Junco insularis* was considered a separate species by most authorities for most of the twentieth century, yet it was lumped with mainland dark-eyed juncos by the American Ornithologists’ Union in 1973 [62] and has remained a subspecific entity (*Junco hyemalis insularis*) until the present [24]. Previous taxonomic assessments emphasized plumage and iris color as taxonomically informative traits, which led to erroneous interpretations: Ridgway [63] found affinities between the Guadalupe junco and the pink-sided junco (his *annectens*), Dwight [64] classified it as a subspecies of the pink-sided junco (*J. mearnsi insularis*), and Miller [22] placed it within the “*oreganus* artenkreiss”. Our genetic results reveal that neither plumage nor iris color are phylogenetically informative in this case. The Guadalupe junco is strongly divergent from mainland juncos in mtDNA sequence, morphology and song, and phylogenetic analysis reveals that it renders “dark-eyed juncos” paraphyletic. We therefore recommend that the Guadalupe junco be reinstated as a full species (*Junco insularis*).

Juncos on Guadalupe Island are critically endangered. Restricted to small patches of cypress (*Cupressus guadalupensis*) and pine (*Pinus contorta*) in the north end of the island, we estimate the total area of suitable junco habitat at just 170 to 210 ha. The cypress groove area was estimated at about 780 ha in expedition reports from the early to mid twentieth century [35], [65] and described already as an “old forest” due to the lack of regeneration caused by the browsing of the introduced goat population. By the time Jehl and Everett [66] visited the island in the early1980’s, the forest had been reduced to a narrow grove of cypresses, increasingly decimated by high mortality due to the old age of most trees. The timely eradication of feral goats in 2007, has since allowed the growth of seedlings and a promising though incipient forest regeneration. However, a forest fire in 2008 reduced prime cypress habitat to less than half, and feral cats and mice still plague the island, so that long-term survival of juncos is anything but guaranteed. Targeted conservation efforts are urgently needed to preserve the unique biodiversity of Guadalupe Island, including the unique Guadalupe junco and its habitat.

### Conclusion

In contrast to prevailing taxonomy, genetic data reveal the Guadalupe junco as an old, well-differentiated lineage, whose similarity to mainland juncos in plumage and eye color is due to evolutionary convergence. Congruent patterns of marked genetic, morphological, and bioacoustic divergence support the recognition of the Guadalupe junco as a well-differentiated evolutionary lineage, demonstrating the limited value of plumage and eye color for inferring evolutionary history and species limits in this genus. Our findings confirm the role of remote islands in driving divergence and speciation, but also their potential role as repositories of ancestral diversity as shown by the richness of the genetic pool and song structure of the Guadalupe junco. Our results also underscore the urgent need to preserve this critically endangered insular bird.

## Methods

### Field Sampling

Junco populations were sampled using mist nets and song recording playbacks to attract individuals to the net when needed. Each individual captured was aged, sexed, and marked with a numbered aluminum band. Morphological measurements were taken (see below), and a blood sample was collected by venipuncture of the sub-brachial vein and stored in lysis buffer at −20°C in the laboratory. After processing, birds were released unharmed at the site of capture. All sampling activities were conducted in compliance with UCLA’s Animal Care and Use Program regulations, and with state and federal scientific collecting permits in the USA, and a special research permit to sample on Guadalupe Island issued by the Secretaria de Medio Ambiente y Recursos Naturales of Mexico (Permit No. SGPA/DGVS/01217/11). Sampling localities for genetic and morphological data (with sample sizes for morphology/genetics specified in parentheses) were as follows: *J. h. insularis* (34/32): Isla Guadalupe, Mexico (N 29.110°, W 118.3267°); *J. h. oreganus* (18/22): Payette National Forest, Idaho (N 45.093°, W 116.635°), Sawtooth National Forest, Idaho (43.898°N, 114.901°W), Malibu, California (N 34.064°, W 118.612°), USA; *J. h. mearnsi* (13/4): Shoshone National Forest, Wyoming (N 43.982°, W 109.515°), USA; *J. h. caniceps* (10/5): Uinta range, Arizona (N 40.805°, W 110.877°), USA; *J. phaeonotus* (34/24): La Cima, D. F. (N 19.253°, W 99.336°), Mexico.

### Genetic Analysis

We extracted genomic DNA from blood samples using a Qiagen DNeasy kit (Qiagen™, Valencia, CA) following the manufacturer's protocol. We amplified two regions of the mtDNA: 349 base pairs (bp) of the hypervariable region I of the control region (CR) using primers LGL2 (L2263, 5′-GGCCACATCAGACAGTCCAT-3′) and H417 (H2607, 5′-AGTAGCTCGGTTCTCGTGAG-3′) [67]; and 640 bp of the cytochrome *c* oxidase I (COI) gene using primers “BirdF1” (5′-TTCTCCAACCACAAAGACATT-3′) and “BirdR1” (5′-CGTGGGAGATAATTCCAAATCCTG-3′) [68]. Primers L16150 (5'-CCTCYAYCWCCARCTCCCAAAGC-3') [69] and “BirdR2” (5'-ACTACATGTGAGATGATTCCGAATCCAG-3') [68] were used instead of LGL2 and “BirdR1” to amplify samples from Guadalupe island. Details on amplification conditions are available from the corresponding author upon request. PCR products were purified with an ethanol precipitation and sequenced in an ABI 3730X automated sequencer. The amplification of nuclear copies of the control region is unlikely since we amplified it together with a coding fragment that was unambiguously translated into its aminoacid sequence. All sequences used in the study have been deposited in GenBank (accessions KC862058–KC862069).

Sequences were aligned and trimmed to equal lengths using Sequencher 4.1.4 (GeneCodes) and the accuracy of variable sites was checked visually on the individual chromatograms. We calculated genetic distances using the concatenation of both mtDNA sequences. Percent divergence was calculated using the number of nucleotide changes between haplotypes (p distances) and correcting for within population variation [70] in Arlequin 3.5.1.2 [71]. We obtained an estimate for divergence time using a standard molecular-clock calibration for coding mtDNA in songbirds of 2.1% per Ma. [31]. In addition, we obtained estimates of divergence time and gene flow between the island and mainland lineages using coalescence analysis of the COI sequences under an isolation-with-migration model as implemented in the program IMa2 [72]. To account for the possibility of multiple nucleotide substitutions per site we used a Hasegawa-Kishino-Yano (HKY) model [73] for the calculations, since an infinite sites model does not apply to our data. Based on preliminary runs, we set prior maxima for divergence time, population size and mutation rate to 25, 20 and 3, respectively. We run ten chains of 10,000,000 steps each, sampling every 100 steps after a 50,000-step burn-in, with heating in a geometric increment model with a term 1 of 0.96 and a term 2 of 0.9. We tracked chain convergence using Tracer v1.5 [74]. Further estimation of divergence times was conducted using BEAST 1.7.2 [75], in MCMC runs of 10,000,000 steps each with sampling every 1,000 steps. We used a strict molecular clock (after ruling out rate variation across branches), and modeled rate variation with a lognormal distribution with a mean of 0.021 and a standard deviation of 0.5.

Nei's [76] unbiased haplotype diversity (*h*) and nucleotide diversity (*π*) values within groups for all three lineages were calculated in Arlequin 3.5. To test for past sudden changes in population size we used Fu's [77] test of neutrality, which detects departures from neutrality in scenarios with biased frequencies of rare alleles or young mutations in non-recombinant sequences. We used Arlequin 3.5 to obtain Fu's F_s_ values, and large and significant negative values of the F_s_ statistic were interpreted as an excess of recent mutations caused by a population expansion.

To establish the relationship between the different haplotypes present in the populations we constructed haplotype networks for both regions and for the concatenated sequence using a median-joining (MJ) algorithm [78] in the program Network 4.6 (fluxus-engineering.com). Haplotypes of the volcano junco (*Junco vulcani*) from Costa Rica, the most divergent junco species (2.82% divergence in COI sequence from the continental radiation lineages and 2.50% from *insularis*), were included for comparison.

### Morphological Analysis

The following morphological measurements were obtained from each bird: unflattened wing length using a ruler to the nearest 0.5 mm; and tail length, tarsus length, bill culmen, exposed bill culmen, bill width and bill depth using a 0.1-mm precision caliper. For details on each measurement see Milá et al. [79]. We measured mass with a digital scale of 0.1-g precision. All measurements were taken by a single observer (BM). To test the significance of the morphological differences between the island and the continental lineages we compared population means for all morphological traits using one-way ANOVA. We also conducted a discriminant function analysis to assess if the three lineages (Guadalupe juncos, mainland dark-eyed juncos, and yellow-eyed juncos) clustered into morphologically differentiated groups. To calculate discriminant functions, variables were transformed using natural logarithms, and mass was linearized using a cubic-root transformation. All analysis were conducted in SPSS 11.5 (SPSS Inc 2002).

### Song Analysis

Song recordings were obtained using a Roland Edirol R-09 stereo digital recorder and a Sennheiser ME66 shotgun microphone and stored as uncompressed wave files. Localities for the recordings were the following: *J. h. insularis* (n = 12): Isla Guadalupe (29.110° N, 118.3267° W), Baja California, Mexico; *J. h. oreganus* (n = 11): Mt. Laguna (32.864° N, 116.442° W), and University of California San Diego (32.876° N, 117.237° W), California, USA; and *J. phaeonotus* (n = 7): San Cristóbal de las Casas (16.733° N, 92.604° W), Chiapas, and Ajusco (19.211°N, 99.283°W), D.F., Mexico.

We analyzed sonograms from song recordings using Raven Pro 1.3 [80]. To measure song variables, we produced a spectrogram for each individual song using a 256 Hann window with a 50% time grid overlap and a discrete Fourier transform (DFT) size of 512 samples. We used Marler and Isaac's [81] definition of “syllable” for junco song, a coherent unit formed by a group of two or more notes, each note being a continuous vocal utterance. Variables measured included maximum and minimum frequencies, peak frequency, song duration, number of different syllables and total number of syllables, from which we obtained a measure of repeated syllables. Mean values for all these measures were calculated for each lineage, and differences were analyzed with SPSS 11.5 by means of one-way ANOVA and discriminant function analysis.
